RETRACTED

# Effect of a Care Bundle Combined with Continuous Positive Airway Pressure in the Postanesthesia Care Unit on Rapid Recovery after Pulmonary Tumor Resection

**DOI:** 10.1155/2021/5906855

**Published:** 2021-10-25

**Authors:** Yongxiang Yan, Jianwei Luo, Liuming Pei, Jianfeng Zeng, Wenchan Yan, Dongni Xu, Shaoman Lin, Xiangbo Wu, Haixuan Zhao, Sihua Liang

**Affiliations:** Surgical Anesthesia Center, Sun Yat-sen Memorial Hospital, Sun Yat-sen University, No. 107, Yanjiang West Road, Yuexiu District, Guangzhou, Guangdong 510120, China

## Abstract

**Objective:**

To study the effect of a care bundle combined with continuous positive airway pressure (CPAP) in the postanesthesia care unit (PACU) on rapid recovery after pulmonary tumor resection.

**Methods:**

A total of 135 patients requiring anesthesia resuscitation after pulmonary tumor resection in our hospital from June 2020 to February 2021 were selected. They were randomly divided into three groups: the PACU experimental group, PACU control group, and operating room resuscitation (OR) group. Subsequently, their intraoperative clinical symptoms, parameters in monitoring postoperative respiratory status, and follow-up results were compared among the three groups.

**Results:**

The PACU experimental group had the highest number of right lesions, while the OR group had the highest intraoperative blood transfusion volume, urine volume, intraoperative colloid volume, intrapulmonary shunt, and intraoperative physician handover rate (*P* < 0.05). Before surgery, serum potassium (K) in the PACU experimental group was significantly higher than that in the OR group but lower than that in the PACU control group (*P* < 0.01). During the time in the PACU, blood partial pressure of oxygen (PO_2_) and oxygen index (OI) levels in the PACU experimental group were significantly higher than those in the other groups (*P* < 0.01). After surgery, total PACU stay time, time from PACU to extubation, and stay after extubation were markedly reduced in the PACU experimental group (*P* < 0.05). The highest number of patients with drainage was found in the PACU experimental group, while the highest number of patients without drainage was found in the PACU control group.

**Conclusion:**

A care bundle combined with CPAP in the PACU can improve the monitoring time of respiratory status and improve blood gas parameters, thus accelerating the postoperative rehabilitation process of patients undergoing pulmonary tumor resection.

## 1. Introduction

In recent years, with the deterioration of the living environment and changes in living habits, the incidence of pulmonary diseases has been increasing yearly. Pulmonary tumor is a common pulmonary disease in clinical practice [1], which is a broad term including two types: benign and malignant. The incidence and mortality of the malignant one account for a large proportion. It is reported that about 500,000 people die of pulmonary tumors each year, so this disease should be paid more attention [2, 3]. Patients with pulmonary tumors show cough, expectoration, decreased body mass, oppression in the chest, and bloody sputum, and even carcinogenesis, which seriously affect the physical and mental health of patients [4]. At present, chemotherapy, radiotherapy, surgery, and molecular-targeted therapy are mainly taken for pulmonary tumors, especially surgery. Conventional thoracotomy is not significantly effective due to large amount of blood loss, severe trauma, and slow postoperative recovery [5].

RETRACTED

As endoscopic technology develops rapidly, widespread application of minimally invasive technology in clinical practice has been achieved, such as video-assisted thoracoscopic surgery (VATS). VATS is an emerging clinical treatment technology, which has little effect on the postoperative activities of patients, resulting in good quality of life of patients and better protection of their body function and immune status. This means that VATS is conducive to further treatment and prognosis and it has a higher clinical application value compared with the traditional thoracotomy [6]. However, patients undergoing VATS for pulmonary tumor resection are usually accompanied by the decline of respiratory function and the increase of lung tissue heterogeneity. These adverse reactions can lead to serious complications during general anesthesia for VATS, such as pulmonary infection, atelectasis, and respiratory failure, further adversely affecting the prognosis [7]. Therefore, it is of great clinical significance to find effective protective measures for anesthesia resuscitation to reduce the incidence of complications after VATS. This paper mainly focused on the safety and clinical effect of care bundles combined with continuous positive airway pressure (CPAP) in the postanesthesia care unit (PACU) on anesthesia resuscitation in patients undergoing VATS for pulmonary tumor resection, in order to provide reference for clinical application.

## 2. Materials and Methods

### 2.1. General Information

This prospective, randomized controlled clinical study recruited 135 patients requiring anesthesia resuscitation after VATS for pulmonary tumor resection in Sun Yat-sen Memorial Hospital, Sun Yat-sen University Hospital between June 2020 and February 2021. A simple randomization method was used to divide the patients into the PACU experimental group (*n* = 50), PACU control group (*n* = 40), and operating room (OR) resuscitation group (*n* = 45). This study was approved by the ethics committee of Sun Yat-sen Memorial Hospital, Sun Yat-sen University (2021-KY-033).

  Inclusion criteria: (1) patients aged 18–85 years who required anesthesia resuscitation after VATS for pulmonary tumor resection; (2) patients with American Society of Anesthesiologists (ASA) I–III; and (3) patients gave informed consent and volunteered for this study
  Exclusion criteria: (1) patients with severe hypertension, heart disease, and obesity; (2) patients with respiratory tract infection; (3) patients with severe cardiovascular malformation or obvious respiratory failure; and (4) patients with ASA IV and above
  Withdrawal criteria: (1) patients dropped out for any reason and withdrew the inform consent; (2) patients occurred serious clinical adverse events or concurrent disease (including severe drug allergic reactions; acute cardiovascular and cerebrovascular accidents; and new malignant arrhythmia), and the investigators believed that it was not in the best interest of the subjects to continue the trial; (3) investigators proposed to terminate the trial; (4) patients who changed to thoracotomy due to specific clinical conditions; and (5) patients who met the exclusion criteria

RETRACTED

### 2.2. Surgical Methods

Preoperative visits were required for proper communication with the patients. During this process, the detailed points and precautions of postoperative resuscitation were explained to the patients to minimize their tension and fear and obtain their trust and cooperation.

In the PACU experimental group, a care bundle was implemented [8]; with body temperature resuscitation and the head of the bed elevated to 60°, the double-lumen endotracheal tube (DLT) was withdrawn to the trachea (24–26 cm), away from the carina of trachea. Subsequently, the ventilator was connected to assist breathing. Intermittent positive pressure ventilation (IPPV) mode was used first, with body weight-based tidal volume, a fraction of inspired oxygen (FiO_2_) of 50%, and an end-tidal carbon dioxide (EtCO_2_) of 35–60 mmHg. Norepinephrine was used to maintain the invasive mean blood pressure (MAP) at 75–90 mmHg. After the recovery of spontaneous breathing, IPPV was converted to the CPAP mode, and changes in parameters such as oxygen flow and pressure in the CPAP machine were examined. According to the patient' clinical symptoms and blood gas parameters, the CPAP parameters were adjusted every 5 min until the patient was awake. When the spontaneous minute ventilation was >5 ml/kg, the DLT was removed, and the patient inhaled air for more than 20 min and then received arterial blood gas analysis before returning to the ward. Patients with Steward score ≥4 could be sent back to the ward.

RETRACTED

In the PACU observation group, the patients were routinely awakened; with the head of the bed elevated to 30° and a warm body temperature, the DLT was not withdrawn to the trachea, and the ventilator was then connected. The synchronized intermittent mandatory ventilation (SIMV) mode was performed first, with tidal volume ranging from 6 to 8 ml/kg standard body weight. After the recovery of spontaneous respiration, the ventilator was removed, and a nasal cannula was connected to the DLT, which provided 4–6 l/min high-flow oxygen. When the patient was fully awake, the DLT was removed, and the patient inhaled air for more than 20 min and then received arterial blood gas analysis before returning to the ward. Patients with Steward score ≥4 could be sent back to the ward.

In the OR group, after the surgery, the patients were placed in the supine position. An anesthesia machine with pressure-controlled ventilation (PCV) was used to assist breathing, with a FiO_2_ of 50% and EtCO_2_ of 35–60 mmHg. After the recovery of spontaneous breathing, the patient turned to the spontaneous breathing mode without withdrawing the DLT to the trachea. When the patient was awake and opened eyes, the DLT was removed, and the patient inhaled air for more than 20 min and then received arterial blood gas analysis before returning to the ward. Patients with Steward score ≥4 could be finally sent back to the ward.

### 2.3. Outcome Measures

1. Comparison of baseline characteristics of patients: age, gender, ASA classification, preoperative complications, hypertension, diabetes, and other complications
2. Comparison of intraoperative clinical symptoms among the three groups: type of surgery (lesion side: left or right), surgery time, anesthetics (desflurane or sevoflurane), with or without application of hormone, blood transfusion volume, colloid volume, intraoperative urine volume, intrapulmonary shunt, and with or without physician handover
3. Comparison of postoperative blood gas parameters among the three groups: including serum K, partial pressure of carbon dioxide (PCO_2_), partial pressure of oxygen (PO_2_), OI, SO_2_, lactic acid (Lac), white blood cell count (WBC), and PH
4. Comparison of postoperative and follow-up results among the three groups: PACU stay time, extubation time, resuscitation time, hospital stay, ejection fraction, with or without application of postoperative negative pressure drainage and the drainage time, the time and dose of chest drainage, and with or without postoperative pleural effusion, pneumothorax, and pneumonia

RETRACTED

### 2.4. Statistical Analysis

Continuous variables were reported as mean ± standard deviation (SD); if normality was assumed, the *t*-test was utilized, and if normality was not assumed, the Kruskal–Wallis test would be used instead. Categorical variables were presented as number and percentage and were compared using the chi-square test or Fisher's exact test (if expected value ≤ 5 was found). A multivariate linear regression model was used to confirm the significance among groups after adjusting the patients' age, preoperative complication, preoperative serum K, and preoperative SO_2_. The estimated means of groups were presented in a bar chart. All analyses were conducted using IBM SPSS V25 (IBM Corporation, Somers, New York). The statistical significance level for all the tests was set at a *P* value <0.05, two-tailed.

## 3. Results

### 3.1. Patients' Basic Characteristics

A total of 135 patients were included in this study, including 50 in the PACU experimental group, 40 in the OR group, and 45 in the PACU control group. The average age was 56.88 ± 9.94 years, and the gender ratio was 1 : 0.99 (male: female = 68 : 67). As indicated in Table 1, the patients' preoperative complications were reported, including hypertension, diabetes mellitus, and other complications. It was found that the OR group had a significantly lower rate of preoperative complications (*P* = 0.046). No significant differences were found in the patients' age, gender, and ASA classification (*P* > 0.05).

### 3.2. Surgery and Intraoperative Information

Table 2 shows the operation related results among groups. There were comparatively more left- and right-side surgeries (lesion side) in PACU control and PACU experimental groups, respectively (*P* = 0.009). No significant differences were found in surgery time (mean: 146.09 ± 56.54 min), anesthetics (desflurane/sevoflurane = 33/102), and hormone use (35.07%) (*P* > 0.05). Comparatively, the OR group was significantly higher in intraoperative transfusion, colloid, urine, intrapulmonary shunt, and physician handover rate (*P* < 0.05).

### 3.3. Patients' Laboratory Results

Laboratory results were recorded preoperatively, postoperatively, and at different time points in the recovery room. As shown in Table 3, the preoperative serum K level in the PACU experimental group was significantly higher than that in the OR group but lower than that in the PACU control group (*P* = 0.004). The blood PO_2_ and OI levels in the recovery room were significantly higher than those in the OR and PACU control groups (*P* < 0.001), while there were no significant differences in blood PCO_2_, SO_2_, Lac, WBC, and PH (*P* > 0.05).

Values are mean ± SD. PACU, postanesthesia care unit; OR, operating room resuscitation; PCO_2_, partial pressure of carbon dioxide; PO_2_, partial pressure of oxygen; OI, oxygen index; Lac, lactic acid; WBC, white blood cell count.

RETRACTED

### 3.4. Postoperative and Follow-Up Results

The postoperative and follow-up results shown in Table 4 indicated that patients in the PACU experimental group had the significantly lowest PACU stay time, including PACU to extubation and stay after extubation (*P* < 0.05). No significance was found in hospital stay, ejection fraction, chest drainage use, postoperative pleural effusion, pneumothorax, and pneumonia (*P* > 0.05). The rate of postoperative negative pressure drainage use was significantly lower in the PACU experimental group (*P* < 0.05); however, no significance was found in average use time (*P* = 0.207).

After adjusting the patients' age, preoperative complication, preoperative serum K, and preoperative SO_2_, the results of PACU stay among groups remained the same as univariate results; that is, the PACU experimental group had the significantly lowest PACU stay time (*P* < 0.05, Figure 1).

## 4. Discussion

In the present study, we investigated the effect of a care bundle combined with CPAP on the effectiveness and safety of rapid recovery after pulmonary tumor resection; the results showed that this strategy could reduce the PACU stay time, including time from PACU to extubation and stay time after extubation, and improve the blood PO_2_ and OI levels of patients. It is indicated that a care bundle combined with CPAP contributes to the rapid recovery after pulmonary tumor resection and has high clinical application value.

In recent years, with the decline of ambient air quality and the aggravation of the population aging, the incidence of pulmonary diseases is increasing yearly, which seriously affects people's quality of life [9]. VATS lobectomy is a common surgical method for treating pulmonary diseases, with the advantages of less trauma, mild pain, high clinical safety, and rapid postoperative recovery [6]. However, this method can further damage the patient's respiratory tract and, thus, increase the risk of complications such as postoperative respiratory tract infection and atelectasis. Therefore, it is necessary to improve postoperative care for the respiratory tract.

One-lung ventilation is a commonly used ventilation mode in anesthesia for thoracic surgery, which allows ventilation of only the nonoperated lung by using an endobronchial tube, thereby improving the surgical field and facilitating surgical procedures [10]. According to the traditional views, the tidal volume of the lung on the ventilated side is 8–10 ml/kg; too small tidal volume may trigger atelectasis, while a relatively large tidal volume can increase ventilation and improve oxygenation [11]. However, large tidal volume and one-lung ventilation cause increased airway pressure, leading to oxidative stress, inflammatory factor release and tissue damage, and a higher rate of complications such as intraoperative hypoxemia and postoperative lung injury [12–14]. Additionally, studies have reported that traditionally large tidal volume ventilation predisposes critically ill patients to ALI/ARDS [15–17].

RETRACTED

The application of the lung protective ventilation strategy (LPVS) can effectively reduce and prevent the abovementioned problems [18]. Traditional ventilation strategies easily lead to alveolar overdistension and ventilator-induced lung injury, such as barotrauma, volutrauma, and shear strain [19]. By contrast, the LPVS avoids lung overexpansion and collapse, reduces mechanical ventilation-induced lung injury and atelectasis, and decreases airway pressure and resistance [10]. Additionally, the LPVS also downregulates the release of inflammatory factors and, therefore, reduces pulmonary and systemic inflammatory injury [10]. Collectively, it is indicated that the LPVS can reduce the incidence of pulmonary dysfunction after lobectomy [16, 20]. Pinheiro de Oliveira et al. [21] showed that the ventilation mode of small tidal volume combined with proper positive end-expiratory pressure (PEEP) could improve mechanical stress, inhibit the production of pulmonary inflammatory mediators, and therefore, effectively reduce postoperative pulmonary complications. In addition, CPAP can be applied for the nonventilated lung to improve oxygenation by expanding the collapsed lung and improving the ventilation/perfusion ratio of the nonventilated lung [22]. Relevant studies have shown that, for patients with spontaneous breathing, CPAP can provide positive pressure in both the inspiratory phase and expiratory phase, which maintains airway dilation, increases lung compliance and gas exchange, and consequently, effectively improves the clinical symptoms and prognosis of patients [23, 24]. These are all consistent with the findings of this study. In this study, compared with the conventional ventilation strategy, postoperative breathing with the LPVS and CPAP mode in patients in the PACU experimental group significantly reduced the length of stay in the PACU and improved the patients' blood PO_2_ and OI levels, which in turn improved postoperative spontaneous breathing.

Pulmonary tumor resection can cause complications and respiratory failure, so nursing intervention is particularly important [25]. Routine nursing interventions are mostly based on clinical experience, without universality and generalization. A care bundle is proposed by the Institute for Healthcare Quality Improvement (IHI) in 2001, which refers to a set of evidence-based interventions, usually 3 to 5 measures, to deal with refractory clinical diseases [26]. These interventions are operable, clear, simple, and feasible, with better effect of their combination compared with the single ones for the treatment and recovery of patients. It means that a care bundle can provide more optimized medical services for patients and improves nursing outcomes [27]. Therefore, CPAP combined with care bundle in this study was more likely to improve the breathing of patients after pulmonary tumor resection with rapid recovery.

RETRACTED

There are some shortcomings in this study. First, the small number of clinical sample cases in each group led to insufficient statistical power of some experimental results. Second, the postoperative follow-up of patients should be extended and more postoperative complications should be counted to provide more bases for the application of CPAP combined with bundle care in the clinical postoperative period.

## 5. Conclusions

In summary, in patients undergoing pulmonary tumor resection, a care bundle combined with CPAP in the PACU has no significant effect on the clinical symptoms of patients, but can improve the respiratory status monitoring time and blood gas parameters and reduce complications. Therefore, this strategy has great advantages in the rapid recovery after pulmonary tumor resection. This study provides a new idea for promoting the development of comfortable medical treatment and also provides a research basis and plan for subsequent derivative research.

## Figures and Tables

**Figure 1:** The PACU stay time among groups after adjusting the patients' age, preoperative complication, preoperative serum (K), and preoperative SO_2_. (a)*P* < 0.05 vs. OR group; (b)*P* < 0.05 vs. PACU control group.

**Table 1:** Basic characteristics of participants.

Parameters	PACU experimental (*n* = 50)	OR (*n* = 40)	PACU control (*n* = 45)	All (*n* = 135)	*P*
Age, years	55.94 ± 10.52	56.00 ± 9.65	58.71 ± 9.50	56.88 ± 9.94	0.321

*Gender*					0.406
Male	22 (44)	20 (50)	26 (57.78)	68 (50.37)	
Female	28 (56)	20 (50)	19 (42.22)	67 (49.63)	

*ASA*					0.262
II	27 (54)	17 (42.5)	17 (37.78)	61 (45.19)	
III	23 (46)	23 (57.5)	28 (62.22)	74 (54.81)	
Preoperative complication	12 (24)	4 (10)	16 (35.56)	32 (23.7)	0.022
Hypertension	8 (16)	2 (5)	11 (24.44)	21 (15.56)	0.047
Diabetes mellitus	3 (6)	2 (5)	3 (6.67)	8 (5.93)	0.947
Other complications	6 (12)	0 (0)	7 (15.56)	13 (9.63)	0.007

Values are mean ± SD or *n* (%). PACU, postanesthesia care unit; OR, operating room resuscitation; ASA, American Society of Anesthesiologists.

RETRACTED

**Table 2:** Surgery and intraoperative information.

Parameters	PACU experimental (*n* = 50)	OR (*n* = 40)	PACU control (*n* = 45)	All (*n* = 135)	*P*
*Surgery type (lesion side)*					0.009
Left	13 (26)	21 (52.5)	24 (53.33)	58 (42.96)	
Right	37 (74)	19 (47.50)	21 (46.67)	77 (57.04)	
Surgery time, min	139.1 ± 53.54	149.1 ± 59.53	151.18 ± 57.55	146.09 ± 56.54	0.541

*Anesthetics*					0.056
Desflurane	11 (22)	15 (37.5)	7 (15.56)	33 (24.44)	
Sevoflurane	39 (78)	25 (62.5)	38 (84.44)	102 (75.56)	

*Hormone use*					0.412
No	36 (72)	24 (61.54)	27 (60)	87 (64.93)	
Yes	14 (28)	15 (38.46)	18 (40)	47 (35.07)	
Transfusion, ml	1149 ± 392.60	1442 ± 459.43	994.67 ± 364.73	1184.37 ± 440.27	≤0.001
Colloid, ml	674 ± 305.6	867.5 ± 338.46	744.44 ± 274.32	754.81 ± 313.79	0.013
Intraoperative urine, ml	567 ± 373.57	802.25 ± 611.85	516.22 ± 280.65	619.78 ± 447.69	0.007
Intrapulmonary shunt, Qs/Qt	31.05 ± 0.47	31.68 ± 0.54	31.6 ± 0.35	31.42 ± 0.54	≤0.001

*Physician handover*					≤0.001
No	32 (64)	8 (20)	37 (82.22)	77 (57.04)	
Yes	18 (36)	32 (80)	8 (17.78)	58 (42.96)	

Values are mean ± SD or *n* (%). PACU, postanesthesia care unit; OR, operating room resuscitation.

**Table 3:** Patients' laboratory results.

Parameters	PACU experimental (*n* = 50)	OR (*n* = 40)	PACU control (*n* = 45)	All (*n* = 135)	*P*
Serum K (preoperative)	3.57 ± 0.35	3.35 ± 0.35	3.61 ± 0.42	3.52 ± 0.39	0.004

*PCO*_*2*_					
Preoperative	40.18 ± 7.24	41.97 ± 6.00	42.88 ± 6.24	41.61 ± 6.62	0.128
Postoperative	47.18 ± 6.43	48.74 ± 7.77	49.11 ± 6.95	48.31 ± 7.05	0.475
Recovery room	44.02 ± 3.42	45.48 ± 4.00	44.12 ± 4.04	44.49 ± 3.84	0.146

*PO*_*2*_					
Preoperative	306.59 ± 142.76	284.15 ± 153.61	275.82 ± 159.81	289.69 ± 151.28	0.593
Postoperative	245.98 ± 132.01	231.64 ± 110.56	227.24 ± 117.1	235.27 ± 119.56	0.790
Recovery room	78.99 ± 9.46	66.49 ± 10.79	68.07 ± 7.02	71.65 ± 10.73	≤0.001
OI (recovery room)	376.12 ± 45.01	316.68 ± 51.35	324.11 ± 33.39	341.17 ± 51.06	≤0.001

*SO*_*2*_					
Preoperative	99.01 ± 1.23	98.55 ± 1.74	98.1 ± 2.43	98.57 ± 1.88	0.063
Postoperative	96.44 ± 13.89	98.57 ± 1.30	98.42 ± 1.51	97.78 ± 8.27	0.477

*Lac*					
Preoperative	1.03 ± 0.61	0.95 ± 0.41	1.01 ± 0.68	1.00 ± 0.57	0.844
Recovery room	1.21 ± 0.76	1.37 ± 0.61	1.36 ± 0.71	1.31 ± 0.70	0.483

*WBC*					
Preoperative	6.83 ± 2.04	6.06 ± 1.50	6.40 ± 1.86	6.46 ± 1.85	0.139
Postoperative	11.32 ± 3.60	11.32 ± 2.99	11.27 ± 3.64	11.30 ± 3.42	0.997
PH (postoperative)	7.34 ± 0.05	7.33 ± 0.06	7.31 ± 0.08	7.33 ± 0.06	0.082

**Table 4:** Postoperative and follow-up results.

Parameters	PACU experimental (*n* = 50)	OR (*n* = 40)	PACU control (*n* = 45)	*P*
PACU stay, min	67.40 ± 17.39	104.83 ± 26.43	100.58 ± 27.59	≤0.001
PACU to extubation	33.16 ± 13.12	41.55 ± 16.98	40.53 ± 19.77	0.033
Stay after extubation	34.24 ± 12.76	63.28 ± 21.31	60.04 ± 20.92	≤0.001
Hospital stay, day	10.98 ± 3.63	11.68 ± 4.80	12.18 ± 6.56	0.518
Ejection fraction, %	69.00 ± 4.24	68.55 ± 4.31	68.40 ± 4.55	0.786

*Postoperative negative pressure drainage use*				0.014
No	10 (20)	4 (10)	1 (2.22)	
Yes	40 (80)	36 (90)	44 (97.78)	
Postoperative negative pressure drainage, days	1.64 ± 0.98	1.73 ± 0.85	1.98 ± 0.99	0.207
Chest drainage use, days	3.08 ± 1.10	3.63 ± 2.69	3.42 ± 1.34	0.341

*Chest drainage, ml*				
Day 0	201.00 ± 202.14	182.18 ± 168.74	192.16 ± 273.53	0.922
Day 1	230.30 ± 137.71	265.83 ± 196.93	258.89 ± 196.76	0.593
Day 2	188.51 ± 97.26	177.05 ± 138.15	160.44 ± 126.39	0.536

*Postoperative pleural effusion, side*				0.870
No	10 (20)	10 (25)	9 (20)	
Left	9 (18)	10 (25)	11 (24.44)	
Right	17 (34)	9 (22.5)	15 (33.33)	
Bilateral	14 (28)	11 (27.5)	10 (22.22)	

*Postoperative pneumothorax, side*				0.270
No	26 (52)	16 (40)	20 (44.44)	
Left	5 (10)	10 (25)	11 (24.44)	
Right	18 (36)	11 (27.5)	11 (24.44)	
Bilateral	1 (2)	3 (7.5)	3 (6.67)	

*Postoperative pneumonia, lesion side*				0.170
No	14 (28)	5 (12.5)	12 (26.67)	
Yes	36 (72)	35 (87.5)	33 (73.33)	

*Postoperative pneumonia, normal side*				0.885
No	28 (56)	21 (52.5)	26 (57.78)	
Yes	22 (44)	19 (47.5)	19 (42.22)	

Values are mean ± SD or *n* (%). PACU, postanesthesia care unit; OR, operating room resuscitation.

RETRACTED

## Data Availability

The data used to support the findings of this study are available from the corresponding authors (Haixuan Zhao and Sihua Liang) upon request.
